The article "Mechanism of Shishiwei Wendan Decoction in the Prevention and Treatment of Lung Adenocarcinoma Using Network Pharmacology and Molecular Docking" was retracted in 2023. Reasons: signs of a paper mill; compromised peer review; unreliable results or conclusions.

# Mechanism of Shishiwei Wendan Decoction in the Prevention and Treatment of Lung Adenocarcinoma Using Network Pharmacology and Molecular Docking

**DOI:** 10.1155/2022/4411054

**Published:** 2022-09-23

**Authors:** Xiaofan Li, Qi Sun, Wenli Ma, Xinzhe Ma, Hongyue Pan, Wei Guo

**Affiliations:** ^1^Ningxia Medical University, China; ^2^Ningxia Minority Medicine Modernization Ministry of Education Key Laboratory, Yinchuan, Ningxia, China

## Abstract

**Objective:**

This study used network pharmacology and molecular docking technology to elucidate the mechanism of action of Shishiwei Wendan Decoction against lung adenocarcinoma.

**Methods:**

By using the world's largest TCM System Pharmacology Database and Analysis Technology Platform (TCMSP) system to conduct in-depth mining analysis and data collection of the main active components of the medicinal components in Shishiwei Wendan Decoction and using the human gene card database (GeneCards), Human Mendelian Inheritance Online System (OMIM), and Human Disease-Related Gene and Mutation Information Database (DisGeNET) to collect the pathogenic targets of lung adenocarcinoma and build a PPI network; for the core drug targets, use GO enrichment analysis and KEGG pathway analysis; use Cytoscape software to build relevant network maps; and use AutoDock to achieve molecular docking.

**Results:**

Shishiwei Wendan Decoction screened 144 active ingredients and 384 drug targets; 7680 lung adenocarcinoma disease targets were obtained, including 380 targets for Shishiwei Wendan Decoction in the treatment of lung adenocarcinoma. GO enrichment analysis demonstrated 2,299 downstream genes, and key target genes were closely related to nutrient levels, membrane rafts, and protein serine/threonine kinase activity; KEGG functional enrichment analysis yielded 179 related pathways, including tumor necrosis factor signaling pathway which is related to the target gene. Molecular docking showed that the core active ingredients and key targets could be well combined.

**Conclusion:**

Through the network pharmacology analysis and molecular docking experiments of Shishiwei Wendan Decoction against lung adenocarcinoma, it is found that Shishiwei Wendan Decoction has multidimensional effects on the treatment of lung adenocarcinoma, and it is the first Shiwei Wendan Decoction to treat lung adenocarcinoma. Decoction in the treatment of lung adenocarcinoma provides biointellectual support and the oretical support.

## 1. Introduction

Lung cancer is now one of the malignant tumors with the highest mortality rate in the world. According to the statistical results released by the World Natural Health Fund and the Global Cancer Research Institute by 2020, the incidence rate ranks second [1]. According to cytological classification, lung cancer can be further subdivided into the following two types, namely, primary small cell lung cancer (SCLC) and primary nonspecific small cell lung cancer (NSCLC) of which the incidence of NSCLC can be as high as about 85% or more [2]. Lung adenocarcinoma is one of the most commonly used human histological subtypes in the diagnosis of NSCLC [3]. The clinical manifestations of early symptoms of lung adenocarcinoma are mostly insidious. The early clinical manifestations of lung adenocarcinoma are relatively insidious, while in the middle and advanced stages, local invasion or distant metastasis occurs, and its treatment effect is poor, and the estimated 5-year survival rate is only 18% [4]. At present, the main treatment methods for lung adenocarcinoma are targeted and immunotherapy [5–7]. Although this therapy has achieved certain clinical efficacy, the population with clinical benefit is still very small [8, 9], and it is not a small number of patients. The 5-year survival rate of patients with lung cancer after treatment is still low (about 20%) [10]. Therefore, there is an urgent need to improve the living conditions of patients and improve the survival rate.

Shishiwei Wendan Decoction is made by Professor Zhu Jinzhong based on Wendan Decoction and combined with his many years of clinical experience. The functions of Ophiopogon japonicus, Solanum lyratum, Acorus tatarinowii Schott, Polygala Radix, Rehmannia glutinosa, and Salvia chinensis [11] are soothing the liver and invigorating the spleen and regulating triple energizer. Yuan Zhu Zhenheng pointed out in “Danxi Heart Method: Phlegm Thirteen”: “Mortal people who have lumps in the middle and lower parts of the body are mostly phlegm,” and the abnormal flow of body fluids will produce phlegm, dampness, and drinking. Therefore, it can be considered that the tumor is caused by the abnormal distribution of body fluids. According to “Lingshu·Benshu,” “Shaoyang belongs to the kidney, and the upper part of the kidney is connected to the lung, so the two are stored.” Among them, the author believes that Shaoyang refers to the gallbladder and the three energizers of Shaoyang, and the Shisiwei Wendan Decoctiom can solve the above problems, Shisiwei Wendan decoction is added on the basis of Wendan Tang. To understand the function of Shisiwei Wendan decoction, we must first understand its basic prescription—Wendan Decoction was first recorded in the book. *“Three Causes Extreme Disease Syndrome Volume Nine Deficiency Syndrome Treatment”* is the name of the book. recorded Shisiwei Wendan decoction: “after the treatment of serious illness, virtual annoyance can not sleep, this gallbladder cold death, this medicine is the main.” This is inherited from Wendan decoction, which is the inheritance of Wendan decoction. Although Wendan decoction is called “warming gallbladder,” but in fact, the treatment focuses on clearing gallbladder and stomach, and its symptoms are more obvious in Zhongjiao, so the most important drugs are regulating qi and resolving phlegm and clearing gallbladder and stomach. Pinellia pinellia is the core medicine of Shiniwei Wendan Decoction; it eliminates dampness and phlegm and treats tumor diseases, etc. Bamboo Ru and Pinellia ternata match, not only resolving phlegm and stomach but also clearing gallbladder heat, making gallbladder and stomach harmonious; Chen Pi Liqi Huatan invigorates spleen dryness and dampness; Fructus Aurantii breaks qi accumulation, resolves phlegm, and dispels ruffian; Poria cocos invigorates the spleen and tranquilizes the heart; licorice Yiqi and middle reconcile various medicines. All kinds of medicines are used together to regulate qi and resolve phlegm, clear gallbladder and stomach, eliminate annoyance, and stop vomiting. Shisiwei Wendan decoction is developed by Professor Zhu Jinzhong on the basis of Wendan decoction and combined with his own clinical experience for many years. In clinical application, it can significantly reduce cough and pain in patients with lung adenocarcinoma. In view of the complex active ingredients in this compound, the current mechanism of Shishiwei Wendan Decoction in the treatment of lung adenocarcinoma is still unclear, and this study was aimed at clarifying the molecular mechanism of its treatment of lung adenocarcinoma.

Network pharmacology is an emerging discipline in recent years. It is a systematic analysis method based on the interaction of diseases, drugs, active ingredients, target genes, and target proteins. The complex synergistic functions and associations also coincide with the notable features of the holistic treatment of modern Chinese medicine and the systemic synergistic treatment of drugs in the treatment of disease processes [12], which can more clearly and intuitively represent the system of the drug itself and its related compounds. The use of network pharmacology can more clearly and intuitively show the complex synergistic relationship between the drug itself and the compound [13, 14]. To this end, this study is aimed at studying the main drugs and their active chemical constituents, traditional Chinese medicine Shishiwei Wendan Decoction used in the treatment of primary lung adenocarcinoma through the technical system of modern network pharmacology technology and drug molecular information docking. The potential target structure and molecular information pathway provide the basis for the further research and development of the safety of the traditional Chinese medicine Shishiwei Wendan Decoction and the evaluation of the clinical use of the drug.

## 2. Methods

### 2.1. Screening of Active Ingredients in Shishiwei Wendan Decoction

Using the TCMSP database (http://tcmspw.com/tcmsp.php), set the oral bioavailability threshold (OB) parameter in the database to ≥30%, the drug similarity threshold (DL) parameter to ≥0.18, and the remaining parameters set as the default value, by adjusting the ADME parameter value to achieve preliminary quantitative screening of the relevant active ingredients of the drug.

### 2.2. Screening of Key Targets for Antilung Adenocarcinoma Effect of Shishiwei Wendan Decoction

The drug active ingredients obtained in 1.1 were imported into Swiss Target Prediction (http://www.swisstargetprediction.ch) to predict relevant anticancer targets. The species parameter was set to “Homo sapiens” to assess the reliability of the predicted results with a confidence threshold.

### 2.3. Lung Adenocarcinoma (LUAD) Disease Target Collection

Setting the keyword to “lung adenocarcinoma” can be obtained from the GeneCards database (https://www.GeneCards.org), the human Mendelian genetic code database (OMIM, http://www.OMIM.org), and human disease-related genes. The corresponding disease target sites were screened in the mutation information database (DisGeNET, Https//http://www.DisGeNET.org). At the same time, the duplicate disease targets obtained by screening were deleted.

### 2.4. Protein-Protein Interaction (PPI) Analysis of the Antilung Adenocarcinoma Target Proteins of Shishiwei Wendan Decoction

The fourteen Wendan Decoctions obtained in 1.3 were entered into the STRING database (https://string-db.org) in turn, and the species was set as “Homo sapiens,” and the confidence was set as >0.7, the main targets were screened, and the protein-protein interaction (PPI) network of the target proteins of Shishiwei Wendan Decoction against lung adenocarcinoma was constructed. Two-dimensional planarization was performed using Cytoscape (version 3.8.2).

### 2.5. Enrichment Analysis

To further study the functions of key target genes, we carried out functional enrichment and analysis. The target of this research project mainly used the R software cluster Profiler 3.18.0 package to realize pathway analysis and Gene Ontology (GO) enrichment analysis based on Kyoto Encyclopedia of Genes and Genomes (KEGG), to find the key to the module. For the common functions and related pathways of a large number of genes in the gene set, the screening conditions were set as *p* < 0.05, counts > 2.

### 2.6. Correlation Network Construction of Shishiwei Wendan Decoction against Lung Adenocarcinoma

Cytoscape (version 3.8.2) software was used to construct a “drug-active ingredient-target-disease network diagram” and a “key target-function regulation network diagram.”

### 2.7. Molecular Docking of the Core Components of Shishiwei Wendan Decoction with Key Targets

The top 5 core active ingredients were calculated by the degree value. First, the 3D Conformer structure of citromitin was downloaded from the PubChem (https://pubchem.ncbi.nlm.nih.gov/) database. Second, download the corresponding crystal structures in the PDB (https://www1.rcsb.org/) database. Then, use AutoDock Vina software to complete the molecular docking experiment. Finally, the interaction between Shishiwei Wendan Decoction and key target proteins was visualized using PyMOL and finally displayed in a two-dimensional plane.

## 3. Results

### 3.1. The Active Ingredients of Shishiwei Wendan Decoction

In TCMSP, the set screening conditions are OB ≥ 30% and DL ≥ 0.18 for screening. The specific screening results are shown in Table 1.

### 3.2. The Active Ingredient Targets of Shishiwei Wendan Decoction

The active ingredients of each drug in 3.1 were imported into the TCMSP database to collect their targets, and 384 targets were obtained after the union was removed and duplicates were removed, as shown in Table 2.

### 3.3. Access to Lung Adenocarcinoma Disease Targets

This study used the GeneCards, DisGeNET, and OMIM databases to obtain disease targets. Using “lung adenocarcinoma” as the key word, the following three databases were firstly searched; secondly, the disease targets retrieved from the three databases were merged, and finally, 7680 lung adenocarcinoma-related disease targets were obtained. Target for subsequent analysis is shown in Table 3.

### 3.4. Obtaining the Key Targets of Shishiwei Wendan Decoction against Lung Adenocarcinoma

In this study, the R language Venn diagram (version 1.6.20) was used to intersect the drug targets obtained above and lung adenocarcinoma (LUAD) disease targets, and 284 key targets were obtained as a result, as shown in Figure 1.

### 3.5. Functional Enrichment Analysis of Key Target Genes in Antilung Adenocarcinoma of Shishiwei Wendan Decoction

#### 3.5.1. GO Analysis Results of Key Targets of Shishiwei Wendan Decoction against Lung Adenocarcinoma

In this study, GO functional annotation was performed on the 284 key target genes described in 3.4, and the biological significance represented by each gene was mined.

Bar graphs were drawn using the R language “enrichplot” (version 1.10.2) to display the GO functional enrichment results (Figure 2(a)). The results showed that in terms of biological process (BP), a total of 1931 terms were obtained, and the key target genes were significantly related to response to nutrient levels, response to oxidative stress and regulation of small molecule metabolic process, etc. It also included cellular response to external stimulus, cellular response to chemical stress and response to drug, and steroid metabolic process. In terms of molecular functions (MF), a total of 189 terms were obtained, and key target genes were significantly related to drug binding, peptide binding, vitamin binding, amide binding, ligand-activated transcription factor activity, etc., including monocarboxylic acid binding, transcription coactivator binding, organic acid binding, carboxylic acid binding, and protein serine/threonine kinase activity. In terms of cellular components (CC), a total of 93 terms were obtained, and key target genes were significantly related to membrane regions, membrane microregions, secretory granule lumen, and cytoplasmic vesicle lumen, including synaptic membrane, postsynaptic membrane, cytosolic large ribosomal subunit, ficolin-1-rich granule, caveola, plasma membrane raft, membrane region, membrane microdomain, and membrane raft.

The ordinate represents the enriched GO term, the length of the bar represents the number of key targets enriched by the GO term, and the color from blue to red represents the reliability of the result from low to high.

#### 3.5.2. KEGG Analysis Results of Key Targets of Shishiwei Wendan Decoction against Lung Adenocarcinoma

In this study, the enrichment analysis of 284 key target genes was carried out with the help of the KEGG database, and 179 related pathways were obtained, and the R language “enrichplot” (version 1.10.2) was used to draw a bubble chart to display the top 15 pathways (Figure 2(b)). It can be seen from the figure that KEGG enrichment results include Th17 cell differentiation, endocrine resistance, prostate cancer, estrogen signaling pathway, chemical carcinogenesis-receptor activation, coronavirus disease-COVID-19, and chemical carcinogenesis-reactive oxygen species, indicating key target Dot genes are significantly associated with tumor necrosis factor signaling pathway, chemical oncogenic-receptor activation, and endocrine resistance.

The bubble volume represents the number of pathway genes, and the color from light blue to red indicates the reliability of the result from low to high.

### 3.6. Key Target Regulatory Network

#### 3.6.1. Key Target-Function Regulatory Network Diagram

We put forward the corresponding key targets of the GO_BP, GO_CC, and GO_MF top 10 terms (the terms of GO_BP, GO_CC, and GO_MF cannot all be displayed) and constructed a key target-function regulatory network diagram and used Cytoscape (version 3.8.2). For visualization, Figure 3(a) is the key target-function network diagram of the terms of GO_BP top 10, which includes 10 terms, 141 key targets, and a total of 398 relationship pairs.  Figure 3(b) is the key target-function network diagram of the terms of GO_MF, which contains 10 terms, 87 key targets, and a total of 182 relationship pairs.  Figure 3(c) is a key target-function network diagram of the terms of GO_CC, which contains 10 terms, 68 key targets, and a total of 207 relationship pairs.

### 3.7. Key Target-Pathway Regulatory Network Diagram

We proposed the KEGG top 20 pathways and their corresponding key targets, constructed a key target-pathway regulatory network diagram, and used Cytoscape (version 3.8.2) to visualize (Figure 4). The network contains 20 KEGG pathways and 139 key targets with a total of 496 relational pairs.

### 3.8. PPI Regulatory Network Diagram of Key Targets

To explore whether there is an interaction between key targets, this study used STRING (https://string-db.org) to construct a PPI network for 284 key targets. The confidence level is 0.7, and the discrete proteins are removed to obtain the interaction network relationship of 349 proteins, including 349 nodes and 4062 edges, as shown in Figure 5(a). The protein network map was beautified using Cytoscape (version 3.8.2), as shown in Figure 5(b). In addition, this study sorted the degrees of genes in the PPI network and screened top 5 genes for subsequent analysis. The top 5 genes ranked by degrees are shown in Table 4. It can be seen that TP53, HSP90AA1, MAPK1, MAPK3, and AKT1 may play a key role in lung adenocarcinoma.

The lines represent the interaction between them; the color represents their degree value, and the darker the color, the higher the degree value, and the more in the core position.

### 3.9. TCM Pharmacological Regulation Network of Key Targets

We proposed the active ingredients corresponding to the five key targets obtained above, constructed a drug-active ingredient-key target gene network key, and used Cytoscape (version 3.8.2). For visualization, as shown in Figure 6, the network contains 10 drugs (Huangqi, Shijianchuan, Banxia, Chenpi, Zhishi, Renshen, Weilingxian, Danggui, Shichangpu, and Maidong), 26 drug active ingredients, 5 key targets, and a total of 73 relationships right.

### 3.10. Molecular Docking Results

First, the protein structures of key targets were obtained from the PDB (https://www1.rcsb.org/) database, and the original small molecules and water molecules were removed (1.5.6). Complete protein hydrogenation and calculate charge. Active ingredient structures were downloaded from the PubChem (https://pubchem.ncbi.nlm.nih.gov/) database and charge-balanced, rotatable bond checks were performed on small molecules using AutoDock Tools. Then, the extent of the docking box is selected according to the receptor active center. Finally, use AutoDock Vina to calculate receptor and ligand docking, and select the structure with the lowest binding free energy (highest binding affinity) in the output. Finally, use PyMOL (version 2.5) software for visualization and beautification. We selected top 5, the core gene of the PPI network, and found the targeted active molecules of these genes in the TCM pharmacological network (the key targets with multiple active molecules are selected according to the comprehensive selection of OB and DL). docking.

### 3.11. Molecular Docking of TP53 and Nobiletin

The 3D conformer structure of nobiletin is shown in Figure 7(a). PDB database downloads the crystal structure of TP53 with PDB ID 6iu7. The molecular docking results are shown in Figure 7(b).

Among them, ALA-1680, LYS-1681, and SER-152 residues have hydrogen bonding interactions with nobiletin molecules. The docking affinity between the active molecule and the protein is -6.2 kcal/mol.

### 3.12. Molecular Docking between HSP90AA1 and Citromitin

The 3D conformer structure of citromitin is shown in Figure 7(c). PDB database downloads the crystal structure of HSP90AA1 with PDB ID 4bqg. The molecular docking results are shown in Figure 7(d).

Among them, the TYR-139 residue has a hydrogen bond interaction with the citromitin molecule. The docking affinity between the active molecule and the protein is -7.4 kcal/mol.

### 3.13. Molecular Docking between MAPK3 and Naringenin

The 3D conformer structure of naringenin is shown in Figure 7(e). PDB database downloads the crystal structure of MAPK3 with PDB ID 2zoq. Molecular docking results are shown in Figure 7(f).

Among them, ASP-123, ASP-184, MET-125, and LYS-131 residues have hydrogen bonding interactions with naringenin molecules. The docking affinity between the active molecule and the protein is -8.7 kcal/mol.

### 3.14. Molecular Docking of AKT1 and Alexandrin

Alexandrin's 3D conformer structure is shown in Figure 7(g). PDB database downloads the crystal structure of AKT1 with PDB ID 5aar. Molecular docking results are shown in Figure 7(h).

Among them, THR-642, LEU-668, LEU-699, GLU-669, and VAL-674 residues have hydrogen bonding interactions with Alexandrin molecules. The docking affinity between the active molecule and the protein is -6.8 kcal/mol.

### 3.15. Molecular Docking of MAPK1 and Quercetin

The 3D conformer structure of quercetin is shown in Figure 7(i). PDB database downloads the crystal structure of MAPK1 with PDB ID 6 g54. The molecular docking results are shown in Figure 7(j).

Among them, ASP-167, MET-108, LYS-114, LYS-54, and ILE-31 residues have hydrogen bonding interactions with quercetin molecules. The docking affinity between the active molecule and the protein is -8.3 kcal/mol.

## 4. Discussion

In this study, the active components and drug targets of fourteen traditional Chinese medicines were predicted by using the online database to predict the disease targets of lung adenocarcinoma, such as Pinellia, Zhuru, and Citrus aurantium, and the following results and conclusions were obtained by bioinformatics analysis: firstly, the active components of all traditional Chinese medicines and their corresponding drug targets of Shishiwei Wendan Decoction were obtained using TCMSP, ETCM, and TCMID databases, and a total of 384 drug targets were obtained. Then, the OMIM, GeneCards and DisGeNET databases were used to obtain the disease targets of lung adenocarcinoma, and a total of 7680 disease targets were obtained.

Through the intersection of drug targets and disease targets, a total of 284 key targets were obtained. The functional enrichment analysis results showed that the key target genes were related to biological processes such as the response to nutrient levels, the response to drugs, and the regulation of fat metabolism. It is significantly related to molecular functions such as drug binding, peptide binding, vitamin binding, and amide binding and cellular components such as membrane region, secretory granule cavity, cytoplasmic vesicle cavity, and membrane microregion. In addition, key target genes are also involved in chemical oncogenic-receptor activation, tumor necrosis factor signaling pathway, endocrine resistance, and interleukin-17 signaling pathway.

In this study, the main active components of Shishiwei Wendan Decoction against lung adenocarcinoma were preliminarily screened by the method of network pharmacology. Experimental studies have found that quercetin can not only reduce the proliferation rate and invasive ability of lung adenocarcinoma cells and promote the apoptosis of A549 cells but also affect tumor progression by increasing the expression of miR-16 and inhibiting the expression of claudin-2 [15, 16]. Chuancheng Pi can significantly reduce the G0/G1 phase cells of A549 cells and reduce the recurrence rate of lung cancer cells. The G2/M phase is blocked, and the proliferation of tumor cells from the cell cycle is inhibited from entering the apoptosis program, thereby effectively improving the development of tumors [17]. According to Liu et al., the inhibitory effect of TNF-*α* affects the expression of Raf-1 and Bcl-2 and then promotes the apoptosis of lung cancer NCI-H460 cells. Yue [19] showed that naringenin has obvious proliferation inhibition and apoptosis promotion effects on A549 cells, and the reaction mechanism may be related to the activation of ROS/P38-MAPK pathway.

The key targets of Shishiwei Wendan Decoction are hsp90aa1, AKT1, MAPK1, MAPK3, and TP53. The hypoxic microenvironment is widespread in tumors, and the Hsp90 pathway, PI3K-Akt signaling pathway, and MAPK signaling pathway are all closely related to the HIF-1 signaling pathway. Studies have found that the phosphatidylinositol 3-kinase (PI3K)/Akt signaling pathway, the upstream pathway of HIF-1, is involved in the regulation of angiogenesis, proliferation, invasion, metastasis, and apoptosis of general tumor cells under hypoxic conditions. The prognosis of cancer patients is closely related [20]. The study found that quercetin can reverse the cisplatin resistance of human A549 lung adenocarcinoma cells by inhibiting EMT and weakening apoptosis through PI3K/Akt pathway [21]. In addition, experiments have shown that some cancer cells can promote the formation and survival of endothelial cell tubes through PI3K/Akt signal pathway, thus changing the microenvironment, which is conducive to tumor growth. This provides a reference for targeted treatment of lung adenocarcinoma [22]. The Hsp90 pathway is a cooperative pathway of HIF-1. Some scholars believe that the binding of Hsp90 to the b HLH-PAS domain of HIF-1*α* under hypoxia can activate HIF-1*α*, indicating that Hsp90 activity has an activating effect on HIF-1*α* [23]. The MAPK pathway includes several key signaling components and phosphorylation events that play a role in tumorigenesis. These activated kinases transmit extracellular signals that regulate cell growth, differentiation, proliferation, apoptosis, and migration functions, due to receptor tyrosine kinases. Abnormal activation of amino acid kinases or gain-of-function mutations, mainly in RAS or RAF genes, lead to alterations in the RAS-RAF-MEK-ERK-MAPK (RAS-MAPK) pathway in human cancers [24]. Stutvoet et al. found that the activity of MAPK pathway plays a key role in the expression of PD-L1 in lung adenocarcinoma induced by EGF and IFN *γ*, However, MAPK pathway does not change the targeted genes, so MAPK may be a target to improve the efficacy of immunotherapy [25]. The extracellular regulated protein kinase (ERK) transduction pathway is the main transduction pathway in the MAPK signaling pathway, and its downstream can also regulate HIF-1. ERK is mainly activated by the abnormally activated Ras target Raf, which in turn activates The phosphorylation of downstream mitogen extracellular kinase (MEK) eventually activates ERK. When stimulated by, for example, mitogen receptors, cytokines, and growth factors, ERK is phosphorylated and then transduced. It enters the nucleus and activates a variety of oncogenes one after another through transcriptional regulation and induction [26].

The research group found that the expression of PRKCZ-AS1 positively regulates the expression of MAPK1 by consulting the literature. Similarly, the expression of MAPK1 is negatively regulated by miR-766-5p expression. Moreover, the binding ability between miR-766-5p and MAPK1 was confirmed. In addition, the knockdown of MAPK1 partially saved the promoting effect of miR-766-5p inhibition on the proliferation and migration of PRKCZ-AS1-transfected lung adenocarcinoma cells. Overall, PRKCZ-AS1 promotes the development of lung adenocarcinoma by upregulating the expression of MAPK1 through spongy miR-766-5p [27]. AKT is a serine-threonine kinase that is overactivated in many cancers, including lung cancer. Using the transgenic mouse model of lung tumorigenesis driven by overexpression of IGF-IR, it was found that the deletion of Akt1 could inhibit the development of lung tumor, while the deletion of Akt2 enhanced the development of lung tumor. Lung tumors that develop without Akt2 are less likely to show discrete nodules and show scattered growth patterns more frequently. RNA sequencing revealed many differentially expressed genes in lung tumors lacking Akt2, among which five genes Actc1, Bpifa1, Mmp2, Ntrk2, and Scgb3a2 were associated with human lung cancer [28]. TP53 mutation is one of the most common mutations in early lung adenocarcinoma (LUAD), which can cause a series of changes in the immune landscape, progression, and clinical outcome of early LUAD. Zeng et al. took the mutant group as a reference. There were significant differences in somatic mutation mRNA-seq miRNA-seq immune infiltration and immunomodulator in patients with mutant LUAD suggesting that TP53 mutation plays a key role in the occurrence and development of lung adenocarcinoma [29].

Then, using Cytoscape (version 3.8.2) to construct the drug-active ingredient key target regulatory network and PPI network, we further counted the degrees, and the top 5 key target genes were TP53, HSP90AA1, MAPK1, MAPK3, and AKT1. Finally, we extracted five key targets and their corresponding active molecules, downloaded protein crystal structures and small molecule 3D structures, and performed molecular docking experiments. The experimental results show that the binding energies of the core components and key targets in Shishiwei Wendan Decoction are all <-5 kcal·mol-1, indicating that there is a strong binding ability between the key target proteins and the drug-active small molecules.

Based on the above analysis, we screened the key targets of all drugs in Shishiwei Wendan Decoction for the treatment of lung adenocarcinoma using an online database. The purpose of this study was to clarify the molecular mechanism of Shishiwei Wendan Decoction in the treatment of lung adenocarcinoma and to provide a theoretical basis and reference value for Shishiwei Wendan Decoction in the treatment of lung adenocarcinoma.

## Figures and Tables

**Figure 1:** Venn diagram of the intersection of drug targets and disease targets. Pink circle represents a disease target for lung adenocarcinoma, and blue circle represents a drug target.

**Figure 2:** (a) GO enrichment bar chart of key target genes. (b) KEGG pathway enrichment bubble chart of key target genes.

**Figure 3:** (a) Key target-GO_BP functional network diagram. (b) Key target-GO_MF functional network diagram. (c) Key target-GO_CC functional network diagram.

**Figure 4:** Regulatory network diagram of key target-pathway.

**Figure 5:** (a) Protein interaction network of initial key targets. (b) Optimizing the protein interaction network of key targets.

**Figure 6:** Drug-active ingredient-key target-disease network.

**Figure 7:** (a) Schematic diagram of the 3D conformer structure of nobiletin. (b) Result of docking between 6iu7 and nobiletin. (c) Schematic diagram of the 3D conformer structure of citromitin. (d) Result of docking between 4bqg and citromitin. (e) Schematic diagram of the 3D conformer structure of naringenin. (f) Result of docking between 2zoq and naringenin. (g) Schematic diagram of the 3D conformer structure of Alexandrin. (h) Docking result of 5aar and Alexandrin. (i) Schematic diagram of the 3D conformer structure of I quercetin. (j) Result of docking between 6g54 and quercetin.

**Table 1:** Active ingredients of Shishiwei Wendan Decoction.

Chinese medicine name	Active ingredient quantity	Chinese medicine name	Active ingredient quantity	Chinese medicine name	Active ingredient quantity	Chinese medicine name	Active ingredient quantity
White vine	15	Poria	34	Iwami wear	16	Ophiopogon japonicus	11
Pinellia	116	Astragalus	87	Wei Lingxian	57	Yuanzhi	12
Tangerine peel	63	Ginseng	190	Schisandra	39	Bamboo Ru	3
Angelica	125	Calamus	105	Citrus aurantium	25	Rehmannia glutinosa	4

**Table 2:** Active ingredient drug targets.

Chinese medicine name	Number of targets	Chinese medicine name	Number of targets	Chinese medicine name	Number of targets	Chinese medicine name	Number of targets
White vine	22	Poria	52	Iwami wear	118	Ophiopogon japonicus	249
Pinellia	227	Astragalus	181	Wei Lingxian	83	Yuanzhi	38
Tangerine peel	102	Ginseng	141	Schisandra	36	Bamboo Ru	10
Angelica	162	Calamus	132	Citrus aurantium	121	Rehmannia glutinosa	17

**Table 3:** Database and disease target data.

Database name	Number of disease targets
GeneCards database (https://www.genecards.org/)	7031
OMIM database (http://www.omim.org/)	66
DisGeNET database (https://www.disgenet.org/search)	2438

**Table 4:** Top 5 key targets for degree ranking of PPI network.

Name	Degree	Neighborhood connectivity	Radiality	Topological coefficient
TP53	71	18.54929577	0.985969457	0.094351825
HSP90AA1	59	19.40677966	0.984512439	0.10205174
MAPK3	51	23.60784314	0.984026766	0.125573634
AKT1	50	24.36	0.983810911	0.130967742
MAPK1	45	23.46666667	0.982515784	0.131835206

## Data Availability

All data, models, and code generated or used during the study appear in the submitted article (Link: https://pan.baidu.com/s/1PJI6KB_SO1REhxR0F4HHpw Fetch Code:7lwc).
